# Risk Prediction of Coronary Artery Stenosis in Patients with Coronary Heart Disease Based on Logistic Regression and Artificial Neural Network

**DOI:** 10.1155/2022/3684700

**Published:** 2022-03-19

**Authors:** Xiaobing Cheng, Weixing Han, Youfeng Liang, Xianhe Lin, Juanjuan Luo, Wansheng Zhong, Dong Chen

**Affiliations:** ^1^Department of Cardiology, The First Affiliated Hospital of Anhui Medical University, Hefei 230022, China; ^2^Department of Cardiology, Hefei Third Clinical College, Anhui Medical University (Hefei Third People's Hospital), Hefei 230022, China; ^3^Department of Pathophysiology, Gannan Medical College, Gannan 341000, China

## Abstract

**Objective:**

Coronary heart disease (CHD) is considered an inflammatory relative disease. This study is aimed at analyzing the health information of serum interferon in CHD based on logistic regression and artificial neural network (ANN) model.

**Method:**

A total of 155 CHD patients diagnosed by coronary angiography in our department from January 2017 to March 2020 were included. All patients were randomly divided into a training set (*n* = 108) and a test set (*n* = 47). Logistic regression and ANN models were constructed using the training set data. The predictive factors of coronary artery stenosis were screened, and the predictive effect of the model was evaluated by using the test set data. All the health information of participants was collected. Expressions of serum IFN-*γ*, MIG, and IP-10 were detected by double antibody sandwich ELISA. Spearman linear correlation analysis determined the relationship between the interferon and degree of stenosis. The logistic regression model was used to evaluate independent risk factors of CHD.

**Result:**

The Spearman correlation analysis showed that the degree of stenosis was positively correlated with serum IFN-*γ*, MIG, and IP-10 levels. The logistic regression analysis and ANN model showed that the MIG and IP-10 were independent predictors of Gensini score: MIG (95% CI: 0.876~0.934, *P* < 0.001) and IP-10 (95% CI: 1.009~1.039, *P* < 0.001). There was no statistically significant difference between the logistic regression and the ANN model (*P* > 0.05).

**Conclusion:**

The logistic regression model and ANN model have similar predictive performance for coronary artery stenosis risk factors in patients with CHD. In patients with CHD, the expression levels of IFN-*γ*, IP-10, and MIG are positively correlated with the degree of stenosis. The IP-10 and MIG are independent risk factors for coronary artery stenosis.

## 1. Introduction

Coronary heart disease (CHD) is a heart disease caused by various degrees of myocardial ischemia, which leads to narrowing or obstruction of blood vessels. The exact mechanism of CHD is not precise, and it is generally believed that its occurrence and development are related to genetic, environmental, and other factors [1–3]. Different types of immune cells play an essential role in forming early atherosclerotic plaque. These immune cells release effector molecules that can accelerate plaque formation. Therefore, atherosclerosis is considered an inflammatory relative disease and is the result of the joint action of various immune factors [4]. Different immune cells can cause multiple immune responses in the vascular wall, and inflammatory cytokines play an essential regulatory role in this process. Among them, T lymphocyte-induced pathological inflammatory response plays a crucial role in the progression of atherosclerosis. Clinical studies have shown that T lymphocytes can be detected at all stages of atherosclerotic plaque formation [5]. Although T lymphocytes act as both proinflammatory and anti-inflammatory cytokines, it is noteworthy that most T lymphocytes in plaques are members of the Th1-cell family [6].

High expression of interferon-*γ* (IFN-*γ*) and its inducible C-X-C chemokinereceptor 3 (CXCR3) are detected in the arterial plaques of patients with coronary heart disease [7–9]. The serum CXCR3 chemokine level is high in patients with hypertension or aortic aneurysm. T-helper-1 (Th1-) related chemokines, including the monokine induced by interference (MIG/CXCL9), interfer-induced protein 10, (IP-10/CXCL10), and interference-induced t-cell alpha chemoattractant (I-TAC/CXCL11), are all induced by IFN-*γ*. These factors play a chemotactic role by interacting with CXCR3. CXCR3 chemokines (including MIG, IP-10, and I-TAC) may play a decisive role in developing atherosclerosis [10, 11]. Those studies have found an independent correlation between serum MIG level and carotid artery plaque, but no studies have reported whether the serum MIG level correlated with coronary artery stenosis.

Logistic regression and artificial neural networks (ANN) have been widely used in the biomedical field [12, 13]. This study is aimed at analyzing the health information of serum interferon in CHD based on logistic regression and the ANN model to provide a new method for the early diagnosis of CHD.

## 2. Material and Methods

### 2.1. General Data

From January 2017 to March 2020, 155 patients with coronary artery disease were randomly selected from the Third People's Hospital of Hefei, hospitalized due to palpitation, chest tightness, chest pain, etc. The diagnostic criteria for CHD were as follows: Patients with typical symptoms; the results of coronary angiography indicated that the lumen stenosis degree of one or more branched of coronary artery > 50%, or the left main artery stenosis degree > 50%. The exclusion criteria are as follows: patients with complicated aortic valve disease, variant angina pectoris, angina pectoris caused by coronary spasm, malignant tumor, infectious disease, autoimmune connective tissue disease, severe liver and kidney dysfunction, and a recent history of surgery or trauma.

A total of 155 patients with CHD were randomly divided into a training set (*n* = 108) and a test set (*n* = 47) according to a 10-fole crossover method. Logistic regression and ANN models were constructed using the training set data. The predictive factors of coronary artery stenosis were screened, and the predictive effect of the model was evaluated by using the test set data. The specific modeling steps are shown in Figure 1.

### 2.2. Serological Examination

For all the enrolled patients, 3 ml peripheral venous blood was extracted on admission or in the morning of the next day. After standing for one hour, the serum was centrifuged at 4000 rotation/min for 15 min. The upper serum was collected, divided into 0.6 ml centrifuge tubes, and placed in the refrigerator at -80°C for storage.

The ELISA was used to detect IFN-*γ* and MIG. The kit was provided by Endogen Company. IP-10 was detected by ELISA, and the kit was supplied by HyCult Biotechnology Company in the Netherlands. All three indicators were tested strictly according to the operation instructions. In addition, routine examinations of liver or renal function, blood lipid, or glucose were performed for all the enrolled patients. Cardiac color ultrasound examination was routinely performed, 12-lead electrocardiogram examination was performed, and the results were strictly recorded. With the written informed consent of all patients, the study plan was approved by the hospital ethics committee.

### 2.3. Grade of Coronary Artery Disease

Coronary angiography was performed with the participation of associate chief physicians qualified for coronary artery disease intervention. According to the number of diseased vessels, coronary angiography was divided into single-, double-, and multivessel diseases. Gensini score is a method to evaluate the severity of coronary artery disease. The more severe the CHD is, the higher the Gensini score.

The degree of lesion of each vessel was quantitatively assessed according to Gensini score: Luminal stenosis ≤ 25% was 1 point, 26% ~50% was 2 points, 51% ~75% was 4 points, 76% ~90% was 8 points, 91% ~99% was 16 points, and 100% was 32 points.

The coronary score coefficients of different segments were different. The score was multiplied by the lesion vessel coefficient, and the final score of the lesion was the sum of the branching scores of each patient. According to Gensini integral, there were three subgroups (Figure 2): 0 ~ 20 points (mild stenosis *n* = 29), 21~40 points (moderate stenosis *n* = 52), and >40 points (moderate stenosis *n* = 27).

### 2.4. Logistic Regression Model

As a logistic regression statistical model in which the most commonly used outcome variable is a dichotomous variable, the general form of logistic regression equation is often expressed as

(1) $$\begin{array}{c} \text{Logit}\left(P\right)=\text{Log}\left(\frac{P}{1-P}\right)=a+b_{1}x_{2}+b_{2}x_{2}+\cdots +b_{m}x_{m}, \end{array}$$

where “*a*” is the constant, *b*_1_, *b*_2_ ⋯ , *b*_*m*_ is a regression coefficient, and *x*_1_, *x*_2_, ⋯*x*_*m*_ is the predictor. Further calculation is expressed as

(2) $$\begin{array}{c} P=\frac{\exp\left(a+b_{1}x_{2}+b_{2}x_{2}+\cdots +b_{m}x_{m}\right)}{1+\exp\left(a+b_{1}x_{2}+b_{2}x_{2}+\cdots +b_{m}x_{m}\right)}. \end{array}$$

The logistic regression was used to determine the risk factors that significantly affected Gensini score.

### 2.5. Artificial Neural Network Model

ANN model is a computer structure and system based on modern neurobiological research, reflecting some human brain characteristics. The ANN uses training and learning methods to compare each neuron's actual output and expected output in the output layer to obtain the error between them. Then, according to the direction of reducing the error, each connection weight is modified from the output layer through each hidden layer and layer by layer and finally returns to the input layer. Thus, the accuracy of input pattern recognition is constantly improved, which can be used to predict the probability of occurrence.

### 2.6. Statistical Method

The data were analyzed by SPSS 23.0 software. Continuous variables were expressed as mean ± standard deviation or median (*P*25, *P*75). The *t*-test and one-way ANOVA were used. When the results of ANOVA showed statistically significant differences between each subgroup, the *q*′ test was used for pairwise comparative analysis of the mean between the groups. The qualitative data were expressed as a percentage (%), and the qualitative data were compared by chi-square test. The Spearman correlation test was used for correlation analysis. Multivariate analysis was performed by logistic regression analysis.

## 3. Result

### 3.1. Comparison of General Clinical Data

There were no significant differences in gender, age, history of drinking and smoking history, history of diabetes and hypertension, body mass index (BMI), total cholesterol, triglyceride, low-density lipoprotein (LDL), non-HDL, myoglobin, IFN -*γ*, MIG, IP-10, with cysteamine acid, and systolic blood pressure between the training set and the test set (*P* > 0.05, Table 1 and Figure 3).

### 3.2. Establishment of the Artificial Neural Network Model

In this study, according to the basic principle of ANN, the data of these influencing factors of 108 CHD patients in the training set were taken as input. The degree of coronary artery ISR corresponding to the patients was taken as output to construct and train the neural network, to realize the prediction effect of the model on coronary artery ISR (Figure 4).

### 3.3. Correlation Analysis of Serum Interferon with Coronary Artery Gensini Score

According to the Gensini score, patients in the training set were divided into three subgroups. The clinical variables correlation analysis showed that the three subgroups were significantly positively related with age, history of DM, hsCRP, BMI, and SBP; negatively correlated with high-density lipoprotein cholesterol; and significantly positively associated with the MIG and IP-10 serum levels (Table 2).

### 3.4. Logistic Regression Model Analysis

The multivariate logistic analysis took Gensini as dependent variables and introduces age, diabetes, IFN-*γ*, MIG, IP-10, and hsCRP into the logistic regression equation. Logistic regression analysis showed that MIG and IP-10 are predictors of Gensini's evaluation. MIG and IP-10 are independent risk factors of coronary artery disease. The results of Logistic regression analysis were shown in Table 3.

### 3.5. Distinction between Logistic Regression and Artificial Neural Network Model

The area under the curve of the logistic regression model in the training set is 0.805 (95% CI: 0.637-0.912), and the area under the curve of the ANN model in the training set is 0.847 (95% CI: 0.651-0.920). The area under the curve of the logistic regression model in the test set is 0.947 (95% *CI*: 0.899-0.963), while that in the ANN model is 0.958 (95% CI: 0.914-0.971). There was no statistically significant difference between the logistic regression and the neural network model (*P* > 0.05) (Figure 5).

## 4. Discussion

In this study, 108 patients with CHD were used as training set to establish logistic regression and ANN models to evaluate the detection factors of coronary artery stenosis and test sets verified the model's validity. According to Gensini integral in the training set, it could be divided into three subgroups, and the Spearman correlation analysis suggested IFN-*γ*, MIG, IP-10, and Gensini integral relationship [14–16]. Logistic regression analysis showed that MIG and IP-10 were independent risk factors for coronary artery stenosis. Therefore, serum IP-10 and MIG levels had potential clinical significance in diagnosing coronary atherosclerosis. Our results are similar to Gaballah et al. [17].

Coronary atherosclerotic heart disease is the leading cause of death and disability in humans worldwide. The pathophysiological mechanism of atherosclerosis remains unclear. Despite years of in-depth research in this field, rapid changes in treatment significantly reduced mortality and improved quality of life. The underlying cause of CHD is atherosclerosis, which is a chronic inflammatory disease. Th1 cells have been reported to be an important determinant of atherosclerosis progression. Their function is to secrete IFN-*γ*, promote the expression of adhesion molecules in endothelial cells and macrophages, and produce cytokines and chemokines [18]. As a decisive regulator of immune function, the IFN-*γ* has also become an essential factor in atherosclerosis [19, 20]. In recent years, many large-scale studies have proved that MIG is involved in atherosclerosis [21, 22]. In this study, IFN-*γ* in the CHD group was significantly higher. The IFN-*γ* also increased with the Gensini score, and the correlation analysis indicated a significant correlation with Gensini [8, 23]. The IFN-*γ* induces MIG and IP-10 secretion, and it has been previously reported that IFN-*γ* induces the co-localization of CXCR3 chemokines in human atherosclerotic plaques. Consistent with the results of this study, the mRNA levels of MIG, IP-10, and IFN-*γ* in CHD patients increased with the increase of Gensini. Th1-related chemokines, including interferon inducing mononuclear factor (MIG/CXCL9), IP-10/CXCL10, and interferon induction of T cell chemotactic factor (I-TAC/CXCL11) will be induced by IFN-*γ*, probably in the process of the development of atherosclerosis play an important role, and vascular disease and atherosclerosis disease are often associated with carotid intimal thickening [24].

Like other IFN-*γ*-induced chemokines, IP-10 can produce different effects by binding CXCR3. These effects include the accumulation of CXCR3 T cells to the site of vascular injury, leading to intimal hyperplasia [25]. Chemokines can selectively induce the release of leukocyte cytokines and endothelial adhesion molecules and promote the accumulation of many inflammatory cells in the lesion site of atherosclerosis, triggering the inflammatory response [26]. At the same time, IP-10 can induce a variety of chemokines in vascular endothelial cells, macrophages, and smooth muscle cells, causing a variety of cascade effects, chemotaxis more inflammatory cells to the lesion site of atherosclerosis, and aggravates tissue damage. Peripheral blood mononuclear cells can produce high concentrations of MIG, IP-10, IFN-*γ*, mRNA and higher proportion of CXCR3+ cells and in mononuclear cell regulation of lymphoid cells in atherosclerotic lesions, migration, and retention using CXCR3 antagonists NBI-74330 treatment in mice, by blocking CXCR3+ T cells from circular migration to atherosclerotic plaques, thereby reducing the formation of atherosclerosis; therefore, these findings suggest that T cell-driven inflammation may play an important role in the progression of human atherosclerosis. In our study, we found that IP-10 was a predictor of Gensini assessment and an independent risk factor of coronary artery disease. In human and mouse models of atherosclerosis, IP-10 is involved in inflammation and angiogenesis in the mechanism of coronary atherosclerosis, making it an attractive biomarker for coronary atherosclerosis. In people of European descent, IP-10 is associated with CHD, hypertension, and symptomatic heart failure [27, 28].

In this study, 155 patients with CHD were included to construct logistic regression and ANN models. The results showed that in the coronary heart disease group, serum MIG and IP-10 levels were positively correlated with Gensini score. The multiple regression showed that MIG and IP-10 were independent risk factors of coronary artery stenosis: MIG (95% CI: 0.876~0.934, *P* < 0.001) and IP-10 (95% CI: 1.009~1.039, *P* < 0.001). In addition, there was no significant difference between the neural network model and logistic regression model (*P* > 0.05). This means that MIG and IP-10 might be specific markers of coronary atherosclerosis. The results of this study have certain clinical significance. In addition, in the training and test sets, there was no statistically significant difference between the logistic regression model and ANN model in the area under the curve (*P* > 0.05). It shows that the logistic regression model and ANN model have good predictive efficiency in CHD.

However, there are several limitations to our study. First, the effectiveness of the prediction model is also affected by the number of variables, types, and sample size. In addition, this study is a single-center study, with fewer cases included and short observation time. In future studies, the number of population cases and multicenter participation will be further increased to further improve risk factors, to determine the application of MIG and IP-10 in coronary artery disease.

## 5. Conclusion

In summary, our results indicate the potential role of serum MIG and IP-10 in the progression of atherosclerosis. These findings also suggested that MIG may be a useful biomarker for the severity of coronary artery disease.

## Figures and Tables

**Figure 1:** Modeling flow chart.

**Figure 2:** Different degrees of coronary artery stenosis. (a) There was no obvious stenosis in the right coronary artery. (b) 50% stenosis in the distal segment of anterior descending artery. (c) 80% stenosis in the middle segment of right coronary artery. (d) 95% stenosis in the middle segment of anterior descending artery, and 95% stenosis in the anterior and middle segments of circumflex branch.

**Figure 3:** Comparison of gender, age, history of drinking and smoking, history of diabetes, and hypertension between training set and test set. There was no statistically significant difference between the two sets (*P* > 0.05).

**Figure 4:** Multilayer perceptron artificial neural network.

**Figure 5:** ROC curves of the logistic regression model and neural network model. (a) Degree of differentiation between the logistic regression model and neural network model in the training set. (b) Test the differentiation between logistic regression model and artificial neural network model.

**Table 1:** Comparison of general clinical data.

Item	Training set (*n* = 108)	Test set (*n* = 47)	*t*/*χ*^2^ value	*P* value
BMI (kg/m^2^)	24.94 ± 2.03	21.34 ± 2.40	2.34	0.643
WC (cm)	85.02 ± 6.54	84.02 ± 8.39	1.68	1.231
TC (mmol/l)	4.78 ± 1.10	4.78 ± 2.01	1.76	1.012
TG (mmol/l)	1.99 ± 1.74	2.10 ± 0.88	1.34	0.810
HDL-C (mmol/l)	0.81 ± 0.26	0.79 ± 0.33	0.40	0.686
LDL-C (mmol/l)	3.21 ± 0.98	3.45 ± 0.78	2.32	0.076
SBP (mmHg)	125.23 ± 14.43	122.51 ± 13.24	1.11	0.271
DBP (mmHg)	85.26 ± 10.89	92.31 ± 10.11	1.67	0.991
Hcy (*μ*mol/l)	14.00 ± 3.26	14.20 ± 3.21	0.35	0.725
hsCRP (mg/l)	1.60 ± 3.31	1.52 ± 3.16	0.14	0.889
IFN-*γ* (pg/ml)	97.5 ± 8.97	96.09 ± 8.31	0.92	0.359
MIG (pg/ml)	103 ± 10.10	104.11 ± 9.31	0.64	0.521
IP-10 (pg/ml)	109 ± 11.01	109.34 ± 10.35	0.18	0.857

Note: BMI: body mass index; WC: waist circumference; TC: total cholesterol; TG: triglyceride; HDL-C: high-density lipoprotein cholesterol; LDL-C: low-density lipoprotein cholesterol; SBP: systolic pressure; DBP: diastolic pressure; hsCRP: hypersensitive C-reactive protein; Hcy: homocysteine; Sdldl-c: small and dense low-density lipoprotein cholesterol; Sdldl-c/LDL-C: ratio of small, dense low-density lipoprotein cholesterol to low-density lipoprotein cholesterol.

**Table 2:** Correlation analysis between Gensini score and clinical variables.

Variable	Mild stenosis		Moderate stenosis		Severe stenosis	
	*r*	*P*	*r*	*P*	*r*	*P*
Age	0.492	<0.001	0.485	<0.001	0.563	<0.001
Male	0.102	0.21	0.087	0.237	0.132	0.322
Smoking	0.034	0.647	0.23	0.231	0.301	0.010
Diabetes	0.561	0.002	0.64	0.002	0.66	0.011
BMI	0.572	0.011	0.670	0.017	0.65	0.012
WC	0.211	0.12	0.302	0.13	0.201	0.003
SBP	0.679	<0.001	0.673	<0.001	0.621	<0.001
HDL-C	-0.173	0.030	-0.164	0.048	-0.201	0.023
hsCRP	0.052	0.541	0.053	0.491	0.544	0.332
IFN-*γ*	0.045	0.323	0.043	0.291	0.213	0.112
MIG	0.607	<0.001	0.794	<0.001	0.787	<0.001
IP-10	0.737	<0.001	0.772	<0.001	0.556	<0.001

**Table 3:** Analysis of risk factors of Gensini score.

Variable	*β*	*P*	OR	95% CI
Age	0.09	0.511	1.009	0.982–1.036
Diabetes	-0.257	0.550	0.774	0.333–1.795
IP-10	0.024	0.001	1.024	1.009–1.039
IFN-*γ*	-0.514	0.343	0.898	0.439–1.81
MIG	-0.100	<0.001	0.904	0.876–0.934
hsCRP	0.108	0.048	1.300	1.007–1.817

## Data Availability

All data analyzed during this study are available from the corresponding author on reasonable request.
